The article "A Dual Discriminator Adversarial Learning Approach for Dental Occlusal Surface Reconstruction" was published in 2022. Journal: J Healthc Eng.

# A Dual Discriminator Adversarial Learning Approach for Dental Occlusal Surface Reconstruction

**DOI:** 10.1155/2022/1933617

**Published:** 2022-04-12

**Authors:** Sukun Tian, Renkai Huang, Zhenyang Li, Luca Fiorenza, Ning Dai, Yuchun Sun, Haifeng Ma

**Affiliations:** ^1^School of Mechanical Engineering, Shandong University, Jinan 250061, China; ^2^School of Mechanical and Electrical Engineering, Jiangxi University of Science and Technology, Ganzhou 341000, China; ^3^Biomedicine Discovery Institute, Monash University, Melbourne, Victoria 3800, Australia; ^4^College of Mechanical and Electrical Engineering, Nanjing University of Aeronautics and Astronautics, Nanjing 210016, China; ^5^Department of Prosthodontics, Peking University School and Hospital of Stomatology, Beijing 100081, China

## Abstract

**Objective:**

Restoring the correct masticatory function of partially edentulous patient is a challenging task primarily due to the complex tooth morphology between individuals. Although some deep learning-based approaches have been proposed for dental restorations, most of them do not consider the influence of dental biological characteristics for the occlusal surface reconstruction. *Description.* In this article, we propose a novel dual discriminator adversarial learning network to address these challenges. In particular, this network architecture integrates two models: a dilated convolutional-based generative model and a dual global-local discriminative model. While the generative model adopts dilated convolution layers to generate a feature representation that preserves clear tissue structure, the dual discriminative model makes use of two discriminators to jointly distinguish whether the input is real or fake. While the global discriminator focuses on the missing teeth and adjacent teeth to assess whether it is coherent as a whole, the local discriminator aims only at the defective teeth to ensure the local consistency of the generated dental crown.

**Results:**

Experiments on 1000 real-world patient dental samples demonstrate the effectiveness of our method. For quantitative comparison, the image quality metrics are used to measure the similarity of the generated occlusal surface, and the root mean square between the generated result and the target crown calculated by our method is 0.114 mm. In qualitative analysis, the proposed approach can generate more reasonable dental biological morphology.

**Conclusion:**

The results demonstrate that our method significantly outperforms the state-of-the-art methods in occlusal surface reconstruction. Importantly, the designed occlusal surface has enough anatomical morphology of natural teeth and superior clinical application value.

The article "A Dual Discriminator Adversarial Learning Approach for Dental Occlusal Surface Reconstruction" was published in 2022. Journal: J Healthc Eng.

## 1. Introduction

Tooth defect and edentulous and dentition defect are common and frequently occurring diseases, which are mainly caused by dental caries, periodontal disease, trauma, and congenital malformation [1, 2]. Among them, dental caries is the main cause of tooth and dentition defects [3]. The *Global Burden of Disease Study* [4] reported that about half of the global population suffers from oral diseases, of which dental defects account for at least 50%. The common types of restorations for defective teeth are full crown and inlay, in which full crown is the main type for large area defect (see Figure 1). However, with the improvement of human oral health awareness, how to make the dental restoration process more intelligent, the dental crown prosthesis more personalized, and fundamentally change the *computer-aided design* (CAD)-based dental crown restoration design method will become a great challenge for dentists.

A CAD-based dental restoration technology has successfully applied digital geometry design and manufacturing into the dental restoration field, which greatly improves the design quality of prosthesis and significantly reduces the work intensity of dentists. Besides, several studies have successfully used finite element analysis (FEA) as a tool for anatomical morphology construction and biomechanical evaluation of the prostheses [5–7]. Although the combination of CAD and prosthetic dentistry leads to many advantages, the existing CAD-driven dental restoration systems all use a standard template tooth database as the design template, which leads to the present situation that the occlusal surface shape is uniform [8, 9]. Therefore, how to make full use of the efficient digital design method and have the design experience of dentists to solve the personalized design of the complex and varied prostheses is the technical bottleneck in the current restoration.

The development of intelligent technologies such as *deep learning* (DL) has brought new solutions for the dental medicine. Compared with the CAD-based restoration method, the empirical data excavated by DL technology are more suitable for the purpose of the dental personalized service. In the process of dental restoration, dentists have accumulated rich experience data on the design of dental crown occlusal surfaces. These occlusal surface shapes contain enough personalized anatomical features, which can meet the requirements of functional dental restoration. Therefore, this will provide basic conditions for the exploration of intelligent dental restoration technology. However, developing an intelligent dental restoration method is challenging: (1) it is lack of large-scale oral clinical database to train an intelligent network for defective teeth restoration [10]; (2) how to design a personalized dental prosthesis satisfying the normal mastication function of patient; and (3) the great difference in tooth morphology among individuals increases the difficulty of training the network model.

The article "A Dual Discriminator Adversarial Learning Approach for Dental Occlusal Surface Reconstruction" was published in 2022. Journal: J Healthc Eng.

Although a personalized design of dental occlusal surface morphology is full of difficulties and challenges, great achievements have been made through the efforts of researchers, which mainly focus on CAD-based ones and DL-oriented ones. In CAD-based methods, researchers try to obtain the desired results by improving and optimizing algorithms. For example, Buchaillard et al. [8] established a statistical model comprising a mean shape and a series of deformation modes to reconstruct the three-dimensional (3D) crown surface. Jiang et al. [3] adopted iterative Laplacian surface editing and mesh stitching to deform a standard template tooth for the defective occlusal surface reconstruction. Fan et al. [11] proposed a dental shape restoration method combining moving least-squares deformation and template feature line matching to reconstruct the crown surface. Zhang et al. [12] proposed a dual-factor constrained deformation framework for defective tooth modeling based on a standard template tooth library. Li et al. [13] developed an extraction algorithm of biological characteristic curve to achieve close matching of dental prosthesis and preparation tooth. It is worth noting that the above methods of manually adjusting the occlusal surface shape of a standard tooth by controlling the deformation point cannot reconstruct the masticatory function of the defective tooth. So, it is still impossible to design a personalized dental prosthesis that is the most suitable for patients. Although the CAD-based manual interactive dental restoration method can restore the shape of the defective tooth, its shortcomings are also obvious: (1) it requires highly skilled and professional operation skills; (2) it integrates into more artificial subjective design ideas of dentist; (3) it is highly dependent on an efficient and robust deformation algorithm; and (4) it requires many intraoral trials and manual grinding for the prosthesis surface, which is another difficulty to be addressed.

In DL-oriented methods, some deep-learned networks have been widely used in dental-related disease diagnosis [14–16] and tooth segmentation [17–19] due to their superior performance, but the research on dental intelligent restoration is relatively lacking. For example, Lee et al. [20] adopted a pre-trained GoogLeNet Inception v3 network for the diagnosis and prediction of dental caries. Moran et al. [21] adopted super-resolution generative adversarial network (SRGAN) model and transfer learning to obtain higher-quality periapical images for the detection of dental caries and periodontal disease. Lian et al. [22] designed an end-to-end 3D convolution network (called MeshSegNet) to automatically label the individual tooth on dental surface. Torosdagli et al. [23] developed fully automated image analysis software for mandible segmentation and anatomical landmarking based on a long short-term memory network. The above methods have achieved impressive results in the corresponding tasks. However, each of them is tailored for special dental tasks, rather than for the occlusal surface reconstruction. Also, the successful application of these methods indicates that DL-oriented methods have great application potential in the field of dental restoration. Recently, a few literature studies have reported the GAN-based frameworks for dental restoration. For example, Hwang et al. [24] applied a Pix2pix [25]-based model for dental crown design. On this basis, Yuan et al. [26] reconstructed the occlusal surface of the missing teeth by introducing perceptive loss and gap distance constraint. Tian et al. [10] proposed a computer-aided deep adversarial-driven dental inlay restoration framework to automatically reconstruct the occlusal surface for a defective tooth. However, these methods only focus on the task of missing small areas of teeth or do not consider the influence of dental biological characteristics (occlusal fingerprint, occlusal groove) on the restoration task, so that the reconstructed occlusal surface by the above methods do not have the anatomical morphology of natural crown.

The article "A Dual Discriminator Adversarial Learning Approach for Dental Occlusal Surface Reconstruction" was published in 2022. Journal: J Healthc Eng.

In this article, we propose a dental occlusal surface reconstruction method using a dual discriminator adversarial network (DentalRecNet) for a partially edentulous patient. The motivation of the proposed method mainly includes two aspects. Firstly, the previous adversarial learning network for medical image completion tasks mainly focuses on the design of the generator, which fails to make full use of the capabilities of discriminator. We propose a dual discrimination strategy, in which the joint decision of two discriminators is applied to minimize the difference between the generated occlusal surface and the ground truth, to improve the reliability of the network. Secondly, aiming at the lack of personalization of occlusal surface shape designed by existing methods, we believe that ensuring the correct occlusal relationship and enough natural anatomical morphological of the generated occlusal surface is the key factor to evaluate the success of restoration treatment. Therefore, we adopt a strategy of gradually increasing the training complexity to restore the complex topography of the tooth surface. Different from the previously mentioned DL-based restoration methods, the proposed DentalRecNet method has several benefits: (1) it is a highly automated solution that no longer requires manual intervention in the occlusal surface design; (2) it is highly efficient to design a tooth prosthesis with enough dental biological characteristics; (3) the reconstruction error of the occlusal surface is relatively small; and (4) it is highly efficient for dentists in oral clinic. For this study, the main contributions are as follows:

1. We propose an adaptive visual distance-based orthogonal projection method for the construction of the standardized tooth database, which can realize the bidirectional reversible mapping between 3D tooth model and depth map.
2. To reconstruct clear tissue structure and details of the defective tooth, an encoder-decoder generator model with dilated convolutional layers is proposed, which can enhance the transfer of effective features. A composite loss function is also designed to guide the network to capture the dental biological characteristics for accurate reconstruction.
3. A dual discriminative strategy is proposed to distinguish fake from real images. The global-local discriminators with different inputs improve the quality of the generated occlusal surface via joint learning by augmenting the decision ability of discriminators via complementary information.
4. Extensive evaluations are conducted on a real-world dental database. Compared with the state-of-the-art methods, the designed network can achieve much better performance regarding both qualitatively and quantitatively.

The article "A Dual Discriminator Adversarial Learning Approach for Dental Occlusal Surface Reconstruction" was published in 2022. Journal: J Healthc Eng.

The rest of the article is organized as follows. The proposed method schemes are described in Section 2.  Section 3 provides the experimental results. Relevant issues are discussed in Section 4. Finally, the conclusion is summarized in Section 5.

## 2. Proposed Methods

The proposed method for reconstructing the defective occlusal surface essentially involves dental depth map generation and dental restoration network, which is graphically shown in Figure 2. In the depth map generation step, an adaptive visual distance-based orthogonal projection method is used to generate the depth maps. In dental restoration step, a dual discriminator network architecture is designed to synthesize missing teeth images, in which two discriminators are learned to distinguish the reconstructed missing crown and whole generated tooth image as real and fake.

### 2.1. Dental Map Generation

The dental depth map has the characteristics of visual image and contains the spatial information of tooth model, which directly reflects the 3D geometric information of occlusal surface. To preserve the geometry information of a dental model, the Euler angle transform and bounding box are firstly used to normalize the 3D tooth model (see Figure 3). The detailed description of the standardized processing is concluded as in Algorithm 1. Then, an image entropy-assisted adaptive visual distance orthogonal projection method is proposed to calculate the dental depth map with more detailed features for network training, and this method can realize the pixel-distance bidirectional reversible mapping.

The detailed steps for calculating depth maps are shown in Algorithm 2. According to the pixel-distance conversion relationship, the dental depth maps are constructed by Algorithm 2. The calculation formula is as follows:

(1) $$\begin{array}{c} pixel=\frac{255\left(h^{\alpha }-d^{\alpha }\right)}{h^{\alpha }}, \end{array}$$

where *α* is an image enhancement factor, and *h* = 6 mm. It is specified that the dental model beyond this plane will not be projected, but will be converted into a pixel value of 0 in the depth map. By adjusting the parameter *α*, dental depth maps with different qualities can be generated.

Image entropy is a statistical form of image features, which reflects the amount of information carried by the image [27]. Therefore, image entropy is used to assist in evaluating the quality of dental depth maps with different *α* values (see Figure 4). The entropy calculation formula is defined as follows:

(2) $$\begin{array}{c} H=-\sum_{t=0}^{m}P_{t}\mathrm{lo}g_{2}P_{t}, \end{array}$$

where *m* is the range of pixel values (0–255), *P*_*t*_ is the probability of the pixel *t* in the image. Based on a large number of experiments, the detailed information of an occlusal surface can be retained when *α* = 2.

### 2.2. Dental Restoration Network

Generative adversarial network (GAN) has made many remarkable achievements in the field of medical image restoration, and its application can avoid the problem of manually designing complex abstract features and inpainting rules [28–32]. Recently, some effective network architectures [10, 33, 34] have been developed to enhance the ability of the adversarial learning, e.g., dual discriminator GAN [35], which simultaneously adopt global and local image content consistency in the discriminative part from different scales. Here, we design a new DL-based occlusal surface reconstruction method by constructing a generative model and a dual discriminative model. As demonstrated in Figure 5, our approach is based on deep convolutional neural network trained for the dental restoration task. A single generative model is used for the missing occlusal surface synthesis, while the two discriminator networks are trained to determine whether or not the occlusal surface has been completed.

The article "A Dual Discriminator Adversarial Learning Approach for Dental Occlusal Surface Reconstruction" was published in 2022. Journal: J Healthc Eng.

### 2.3. Deep Generative Model

Due to the excellent performance of the encoder-decoder architecture in a variety of medical image analysis tasks [36, 37], we adopt a similar network architecture as a generator, which allows for improved computational efficiency by initially decreasing the resolution before further processing the image. Then, the output is restored to the original resolution image using deconvolution (Dconv.) layers. Unlike other pooling-based architectures to decrease image resolution, our network model uses a convolution operation with fractional strides (¼) to decrease the resolution twice, which can generate an occlusal surface with the clear tissue structure in the missing teeth. As shown in Figure 5(a), the network is formed by layers in which a bank of filters is convoluted with the input images to produce an occlusal surface image. After each convolution (Conv.) layer, except the last one, a batch normalization (BN) and a rectified linear unit (ReLU) activation function are added, while the output layer consists of a Conv. layer with a sigmoid function to normalize the output to the [0, 1] range.

To ensure that the network can handle complicated occlusal surface reconstruction, we add dilated convolutional layers [38] to enhance the learning ability of the network, which mainly uses kernels that are spread out and allows each output pixel to be calculated with a much larger input area. Different from the general connection, the dilated convolutional layers concatenate the previous feature maps to subsequent outputs in the channel, respectively, as illustrated in Figure 6. Moreover, the dilated convolution layer obtains fine-grained structural information and expands receptive fields for efficient feature representation. To reconstruct clearer tissue structure of the dental occlusal surface, the different dilation rates are set to obtain receptive fields with suitable scales. In addition, this connection allows each feature map to undergo several convolution operations at different dilation rates, to capture different types of feature information. The feature mapping of each layer is integrated into the output of the last dilated convolution, so that the generative model can extract more effective and richer biological characteristics.

More specifically, if one 2D layer is an *i*th channel *h*_*i*_ × *w*_*i*_ image and the next layer is an *i*+1th channel *h*_1_+1 × *w*_*i*_+1 image, the dilated convolution operator can be written for each pixel as follows:

(3) $$\begin{array}{c} y=F\left(b+\sum_{i=-k_{h+1}}^{k_{h+1}}\sum_{j=-k_{w+1}}^{k_{w+1}}M_{k_{h+1}+i,k_{w+1}+j}x_{\lambda i,\lambda j}\right), \end{array}$$

where *k*_*n*_+1=*k*_*n*_ − 1/2 and *k*_*w*_+1=(*k*_*w*_ − 2)/2 are the kernel width and height, respectively; *y* and *x* are the pixel component of the input and the output of the layer; *F*(·) denotes a component-wise nonlinear transfer function; *b* is a bias vector; *M* represents *i* + 1-by-*i* matrices of the kernel; and *λ* is the dilation factor.

The article "A Dual Discriminator Adversarial Learning Approach for Dental Occlusal Surface Reconstruction" was published in 2022. Journal: J Healthc Eng.

### 2.4. Global-Local Discriminative Models

Relative to a remarkable generative model, a powerful discriminator is somehow more significant for training a good restoration network. To encourage more realistic crown details, we adopt a dual discriminator network as GAN discriminator to differentiate high-resolution real and synthesized dental images. During the training, both global discriminator *D*_*G*_ and local discriminator *D*_*L*_ share the same generator *G* but examine its output in different ways. The global discriminator *D*_*G*_ takes preparation teeth and adjacent teeth as the input, while the local discriminator *D*_*L*_ takes only the preparation teeth as the input. An overview of two discriminators can be seen in Figures 5(b) and 5(c). Given a preparation tooth with adjacent teeth *x*_1_, and the corresponding target crown with adjacent teeth *z*_1_, the objective function of the adversarial learning is formulated as follows:

(4) $$\begin{array}{c} L_{D_{G}}\left(G,D_{G}\right)=E_{x_{1},c_{1},c_{2},d,z_{1}}\left[\log\;D_{G}\left(x_{1},c_{1},c_{2},d,z_{1}\right)\right]+E_{x_{1},c_{1},c_{2},d}\left[\log\left(1-D_{G}\left(G\left(x_{1},c_{1},c_{2},d\right)\right)\right)\right], \end{array}$$

where *c*_1_ denotes the opposing tooth, *c*_2_ denotes the dental biological morphology (occlusal fingerprint and occlusal groove), and *d* represents the gap distance between two jaws. The generator *G* makes effort to minimize this objective function, while global discriminator *D*_*G*_ tries to maximize it by min_*G*_max_*D*_*G*_,*D*_*L*__*L*_*D*_*G*__(*G*, *D*_*k*_). Similarly, the objective function of the second discriminator is formulated as follows:

(5) $$\begin{array}{c} L_{D_{L}}\left(G,D_{L}\right)=E_{x_{1}^{\prime },c_{1}^{\prime },c_{3},d,z_{1}^{\prime }}\left[\log\;D_{L}\left(x_{1}^{\prime },c_{1}^{\prime },c_{3},d,z_{1}^{\prime }\right)\right]+E_{x_{1}^{\prime },c_{1}^{\prime },c_{3},d}\left[\log\left(1-D_{L}\left(G\left(x_{1}^{\prime },c_{1}^{\prime },c_{3},d\right)\right)\right)\right], \end{array}$$

where *x*′_1_ denotes a preparation tooth, *z*′_1_ is the corresponding target crown, *c*′_1_ represents the opposing tooth of the preparation tooth, and *c*_3_ represents occlusal groove of the target crown.

The article "A Dual Discriminator Adversarial Learning Approach for Dental Occlusal Surface Reconstruction" was published in 2022. Journal: J Healthc Eng.

Effective adversarial training is necessary to ensure the quality of the occlusal surface reconstruction. Therefore, the global discriminator takes the convolutional filter with the size of 5 × 5 and the stride with the value of 2. The fundamental idea is that the generated occlusal surface should not only be realistic, but also consistent with the adjacent teeth shape. Local discriminator follows the same structure pattern, which consists of five convolutional layers and a fully connected layer. It determines whether the reconstructed occlusal surface on the missing tooth location is real or not. Finally, the outputs of two discriminators are fused together by a concatenation layer, which predicts a continuous value corresponding to the probability of the dental image being real. Our ultimate goal is to learn the generator network conditioned on the preparation tooth and the dental biological morphology. Then, the different scale images generated by generator *G* are encouraged to be realistic enough to fool the two discriminators *D*_*G*_ and *D*_*L*_. Therefore, the adversarial learning problem becomes a multi-objective learning problem, which is defined as follows:

(6) $$\begin{array}{c} \underset{G}{\min}\underset{D_{G},D_{L}}{\max}\sum_{k=G,L}L_{GAN}\left(G,D_{k}\right). \end{array}$$

### 2.5. Loss Function

To train the network to reconstruct the realistic dental crown, the adversarial loss (*L*_*adv*_) of GAN in (6) is improved by adding a perceptual loss (*L*_*per*_), a L1 loss (*L*_*L*1_), and a mean-squared error (*L*_*mse*_). Using the mixture of the four loss functions allows the stable training of the occlusal surface reconstruction network. Below, we will explain the reason why we choose these loss terms.

The mean-squared error (MSE) is one of the most widely used fidelity measuring metrics in medical image analysis research. It evaluates the difference between the generated dental image *G*(*x*) and the corresponding target dental crown *z* at the pixel-wise level and objectively quantifies the strength of the error signal [38]. So, we use MSE loss to stabilize the training:

(7) $$\begin{array}{c} L_{mse}=E_{x,z}\left[{\left\|G\left(x\right)-z\right\|}_{F}^{2}\right], \end{array}$$

where ||·||_*F*_ represents the Frobenius norm.

In contrast to MSE loss, perceptual loss evaluates two dental images at the feature level rather than at the pixel level, which helps to preserve the details of the generated occlusal surface and make it clearer in terms of the structure. Therefore, the perceptual loss is added to the training of the network to further improve the ability to reconstruct the biomorphic features of missing teeth. The perceptual loss can be expressed as follows:

(8) $$\begin{array}{c} L_{\mathrm{per}}=E_{x,z}\left[\frac{1}{\mathrm{CHW}}\sum_{i=1}^{N}{\left\|h_{i}\left(z\right)-h_{i}\left(G\left(x\right)\right)\right\|}_{1}\right], \end{array}$$

where ||·||_1_ represents the *L*1 norm, *h*_*i*_ indicates the feature map obtained by the *i*th convolution layer, and *C*, *H*, and *W* stand for the width, height, and depth of the feature space, respectively.

The article "A Dual Discriminator Adversarial Learning Approach for Dental Occlusal Surface Reconstruction" was published in 2022. Journal: J Healthc Eng.

The total loss function is a weighted sum of the above losses, which is formulated as follows:

(9) $$\begin{array}{c} L_{total}=L_{\mathrm{adv}}+\lambda_{L1}L_{L1}+\lambda_{mse}L_{\mathrm{mse}}+\lambda_{per}L_{\mathrm{per}}, \end{array}$$

where *λ*_*L*1_, *λ*_*mse*_, and *λ*_*per*_ are three constant weighting factors.

## 3. Experiment Results

### 3.1. Dental Dataset

Since we do not have enough manpower and professional knowledge of stomatology to collect the damaged and repaired tooth of patients, it is difficult to build up a sufficient number of dental database for network training by ourselves. In view of this situation, this project is cooperated with *Peking University Hospital of Stomatology*, which provides us with manually designed tooth preparation and extracted dental biological morphology. Many studies have reported that the caries rate of mandibular first molar is the highest [3, 10, 12], so we selected patients with defective #46 or #36 teeth as research object (see Figure 7). The 3D digital dental dataset is collected from subject's dental plaster model by 3Shape dental scanner (D700, Denmark), and the dental samples are randomly divided into three parts: 850 for training, 90 for validating, and the remaining 60 dental samples for testing.

### 3.2. Implementation

The proposed dental restoration network is based on *TensorFlow* framework [39], and all experiments are performed on an *Intel (R) Platinum* 8168 CPU @ 2.70 GHz machine running Windows 10 with 128 GB RAM and *GeForce GTX 1080Ti* GPU. To train the model, we optimize the network using the Adam solver with the following hyper-parameters: *λ*_L1_ = 100, *λ*_*mse*_ = 50, *λ*_*per*_ = 50, *β*_1_ = 0.5, *β*_2_ = 0.999, learning rate = 0.0002, and all *ReLUs* in the network with slope 0.2.

### 3.3. Ablation Study

#### 3.3.1. Loss Function Results

To make all the objective constraint functions play the expected role and give full play to the characteristics of the function itself, we adopt a strategy to gradually increase the training complexity on the basis of ensuring sufficient gradient update in the early stage of training. The training process is split into three phases: first, the generator network is trained with occlusion spatial constraint, dental biological morphology constraint, and the *L*1 loss to yield a basic occlusal surface (marked as Stage I). Afterwards, the generator network is fixed and the two discriminators are trained from scratch with MSE loss and perceptual loss (marked as Stage II). Finally, the generator network and a dual discriminator network are trained jointly until the end of the whole training (marked as Stage III).  Figure 8 shows two typical restoration samples with three different settings, one of which is #36 tooth and the other is #46 tooth. The occlusal surface shape generated on the preparation teeth is very close to the object shape when the training reaches the third stage.

The article "A Dual Discriminator Adversarial Learning Approach for Dental Occlusal Surface Reconstruction" was published in 2022. Journal: J Healthc Eng.

In addition to visual results (see Figure 8), three metrics are used to evaluate the performance of occlusal surface generation task. The peak signal-to-noise ratio (PSNR) has become common method to evaluate the quality of compressed and inpainted images [40], which provides pixel-based errors for the processed image towards the target image. The second one is the feature similarity index measure (FSIM) [10], which directly measures the difference in pixel values at the local position of two images. The third metric is the structural similarity index measure (SSIM) [41] that evaluates the holistic structural similarity between two images.  Table 1 provides the average performance of different settings. We can see that the average PSNR value obtained by Stage III increases by 6.431 dB compared with Stage I. In addition, FSIM increases from 0.961 to 0.993, showing the capability of the proposed network to measure the difference in pixel values at the local position of the generated occlusal surface image and target image. The improvement in terms of SSIM, which increases from 0.933 to 0.985, demonstrates the strong capacity of the proposed network in maintaining occlusal surface structures.

During the training process, the *L*1 loss (*L*_*L*1_), the mean-squared error (*L*_*mse*_), the perceptual loss (*L*_*per*_), and the adversarial loss (*L*_*adv*_) in each iteration are recorded for monitoring the convergence of DentalRecNet. To evaluate the performance of each loss used in the proposed DentalRecNet, we adopt a staged training method during the network training process.  Figure 9 plots the training loss of our network versus the number of iterations, which shows that the network achieves a stable decrease in the loss value.

### 3.4. Parameter Selection Results

By adjusting the enhancement factor *α*, we further evaluate the influence of the generated dental image quality of the proposed method, with the results shown in Figure 10. It can be seen that the enhancement factor 2.0 achieves the best performance than the other six parameters, which is consistent with the conclusion as shown in Figure 4. Therefore, the dental depth map obtained by these parameters is used to train DentalRecNet in the experiment.

The article "A Dual Discriminator Adversarial Learning Approach for Dental Occlusal Surface Reconstruction" was published in 2022. Journal: J Healthc Eng.

### 3.5. Effectiveness of the Dilated Convolutional Layers

We then conduct a set of experiments to validate the effectiveness of the dilated convolutional layers used in DentalRecNet. In these experiments, we use the general convolutional layers (General Conv.) to replace the dilated convolutional layers (Dilated Conv.) to construct the generator for the result analysis. According to the gray distance mapping relationship, the 3D model of dental depth image is obtained using an adaptive mesh reconstruction method based on point cloud density.  Figure 11 shows a typical restoration sample with two different settings. It is observed that Dilated Conv.-based generator achieves the better results compared with General Conv.-based generator. In particular, the occlusal fingerprint distribution generated by the DentalRecNet is relatively close to the ground truth sample.

To evaluate the quality of the occlusal surface, the deviation between the generated result and the target crown is calculated under the constraint of the adjacent teeth. As shown in Figure 11, we can see that the standard deviation (SD) value and root-mean-square (RMS) value obtained by the proposed generator decrease by 0.078 mm and 0.081 mm compared with the General Conv.-based generator, respectively.

### 3.6. Comparison Results with State-of-the-Art Methods

#### 3.6.1. Qualitative Results

In this section, we compare the proposed method with five representative GAN-based methods, including Pix2pix [25], CrownDesNet [24], Dental-GAN [27], DAIS [10], and GL-GAN [34]. Pix2pix is a conditional GAN model, which is used to learn a translation function from input to output image domain with paired training samples. CrownDesNet is a dental crown design network, which is used to learn the mapping between the prepared jaw and the dentist-designed jaw with paired training samples. Dental-GAN is a dental crown restoration network based on Pix2pix, which generates more realistic occlusal surface images by adding the perceptual loss and occlusal groove filter loss functions. DAIS is dental inlay restoration network, which is composed of a generative model with a specially designed training strategy, a dual local-global discriminative model, and a parsing model. GL-GAN consists of a completion network based on a fully convolutional network and a global-local context discriminator.

The article "A Dual Discriminator Adversarial Learning Approach for Dental Occlusal Surface Reconstruction" was published in 2022. Journal: J Healthc Eng.

According to the pixel-distance bidirectional reversible mapping relationship, the 3D dental occlusal surface is reconstructed from a generated image using the mesh reconstruction method based on region growth. We visually compare the reconstructed results with three typical examples presented in Figure 12 and provide the occlusal fingerprint (seagreen color) extracted by a dentist. It can be seen that the occlusal surfaces generated by Pix2pix and CrownDesNet have fewer occlusal fingerprints or a smoother occlusal groove. Dental-GAN and GL-GAN show better performance compared with CrownDesNet. The distributions of the occlusal fingerprints generated by DAIS are more reasonable than for the other methods. The reconstructed results of DentalRecNet are relatively close to a natural tooth crown, especially for the occlusal fingerprint distribution and the occlusal groove characteristic.

In addition, an experimental case (see Figure 13) has been added to further verify the effectiveness of the proposed method. In theory, the left teeth (#36) and right teeth (#46) of a person are symmetrical. As can be seen, the dental crown model designed by our method is more personalized than the crown designed by dentist. The dental prosthesis generated by the proposed DentalRecNet model is morphologically similar to the contralateral tooth, which further shows that our method has superior clinical applicability.

#### 3.6.2. Quantitative Results

Quantitative comparisons in terms of PSNR, FSIM, and SSIM are summarized in Table 2. It can be seen that Pix2pix, CrownDesNet, and GL-GAN have lower values for PSNR, FSIM, and SSIM, indicating that it cannot accurately reconstruct more biological characteristics of the occlusal surface. Compared with the crown design network (CrownDesNet), Dental-GAN and DAIS can obtain better results. At the same time, DentalRecNet significantly outperforms the other five methods, which is consistent with the visual results as shown in Figure 12. Therefore, the practical utility of DentalRecNet for automated occlusal surface reconstructing on the missing tooth is further demonstrated.

In addition, we further evaluate the effectiveness of the proposed method with the other existing methods intuitively. The RMS value between the generated occlusal surface and the natural tooth crown is measured, and a series of statistical analyses are performed on the similarity measurement results (see Figure 14). It can be seen that the results obtained by our method are significantly better than other methods. In particular, the detection error by DentalRecNet is 0.114 mm, while the detection error by the optimal DAIS in other methods is 0.164 mm. Furthermore, a one-way ANOVA test is conducted to evaluate the similarity of the deviation measurements between the generated and object tooth crowns. For these six methods, we find a statistically significant difference in deviation measurements (*p* ≪ 1*e* − 3). Similarly, we find a statistically significant difference between DentalRecNet and the other five methods (*p* ≪ 1*e* − 3) using the Kruskal–Wallis test.

The article "A Dual Discriminator Adversarial Learning Approach for Dental Occlusal Surface Reconstruction" was published in 2022. Journal: J Healthc Eng.

## 4. Discussion

Reconstructing the correct spatial occlusal contact relationship of the defective tooth is the basis for evaluating the successful restoration and for maintaining oral health. Considering that each tooth has the same characteristic shape as its standard tooth of the same name, bionic geometry morphology design-based methods tend to adopt the standard dental to design crown [12, 42]. In the process of crown design, occlusal fingerprint is necessary to fully reflect the functional characteristics of the occlusal surface since it provides reference for the position and direction of the correct occlusal contacts [43]. If the occlusal fingerprint distribution is not considered during the design process, there will be a large amount of unreasonable interference areas on the designed crown. This becomes particularly important since occlusal fingerprint helps in dissipating tensile stresses over the dental crown [44]. The unique occlusal groove characteristics of the dental crown determine the direction of food flow and masticatory efficiency during the chewing process, which is also used as a criterion to evaluate the success of the dental restoration. Thus, oral restorations that do not consider occlusal fingerprint and occlusal groove may favor the occurrence of enamel crack and other disruptive processes.

To verify the effectiveness of the proposed DentalRecNet, we compare it with two representative GAN models [25, 34] and three GAN-based dental restoration methods [10, 24, 27]. The visual example results are shown in Figure 12. Compared with Pix2pix and GL-GAN, DentalRecNet can obtain more realistic occlusal surface morphology, and the dental biological characteristics (occlusal fingerprint, occlusal groove) are closer to natural teeth. In addition, our method is also superior to the existing state-of-the-art dental restoration methods, and it can generate more and suitable functional feature areas on the occlusal surface.

Having introduced an approach to represent occlusal surface morphology using depth map, we solve the problem that it is difficult to reconstruct the occlusal surface, which satisfies the normal masticatory function and natural shape based on the template tooth. Despite appearing simple at first glance, bionic geometry morphology design-based method requires large numbers of sample teeth and manual interactions; one would need to define what is the most suitable occlusal surface and how many feature points are selected, when the occlusal surface design is completed, and how to quantify the occlusal functional characteristics area. To find such evaluation criteria and determine the relevant parameters, one in principle needs to analyze the designed crown models (thousands or even more) of 32 tooth types. These design rules would presumably be different across types and consequently lead to different types of teeth are used with different design standards and parameters. However, it has been proved that all these challenges can be solved through deep learning network. These multilevel network architectures are trained by large-scale data to obtain numerous more representative feature information. Hence, instead of manual deformation for each specific tooth, we collect large numbers of cases that specify the constraint condition (opposing jaw, gap distances, occlusal groove, and occlusal fingerprint) for a given input (preparation tooth) and then minimize loss function, which quantifies the statistical differences between the features of the object image and the generated image. Through this minimization, the weights of the network are optimized to improve its generation ability. In particular, deep network has the ability to automatically learn high-level and more discriminative features from the sample dataset, and GAN has achieved outstanding results in synthesizing realistic images by learning complex generative model [23, 45, 46].

The article "A Dual Discriminator Adversarial Learning Approach for Dental Occlusal Surface Reconstruction" was published in 2022. Journal: J Healthc Eng.

## 5. Conclusions

In this article, a novel dental occlusal surface reconstruction model for masticatory function restoration from partially edentulous patient is proposed, which includes a dilated convolutional-based generative model and a dual discriminative model. In particular, the dilated convolution structure is exploited in the generative model to obtain discriminative feature representations and preserve more fine-grained biological feature information for accurate reconstruction. The dual global-local discriminative model attempts to enhance the discrimination ability for a better decision, which optimizes the generative model more effectively with two separate yet complementary discriminators. Experimental results demonstrate that, under the same conditions, the proposed approach outperforms recent advances on the real-world dental database. In particular, the detection error by our method is 0.114 mm, while the optimal detection error of other methods is 0.164 mm. Meanwhile, it also verified that the proposed DentalRecNet has potential application value as an intelligent and personalized dental restoration method. Importantly, the proposed method realizes the transformation of prosthesis from geometric shape design to functional characteristic design.

The article "A Dual Discriminator Adversarial Learning Approach for Dental Occlusal Surface Reconstruction" was published in 2022. Journal: J Healthc Eng.

Although DentalRecNet has achieved the most advanced performance in solving the challenging problem of personalized dental occlusal surface reconstruction, several technical issues should be still considered in the future. (1) In current DentalRecNet, the dental depth images are used for network training, which requires an additional post-processing process to design a 3D dental crown. Therefore, an end-to-end solution for dental crown reconstruction can be explored to further simplify the restoration process; (2) the current training dataset contains only mandibular first molar (#36 or #46) with the highest tooth defect rate. Considering the randomness of defective teeth, it is necessary to establish a larger dataset containing more tooth types, which can further improve the clinical performance of DentalRecNet.

## Figures and Tables

**Figure 1:** Typical 3D dental crown examples. The first row shows the matching relationship between the dental crown and the preparation teeth, and the second row provides the related physical models of the dental crown.

**Figure 2:** Overall flowchart of the proposed DentalRecNet. Firstly, the dental depth images are calculated from the 3D tooth models by an orthogonal projection method. Then, dental restoration network based on an encoding-decoding generator and a global-local discriminator is employed to reconstruct the missing occlusal surface.

**Figure 3:** Standardized processing of tooth model posture.

**Figure 4:** Entropy values of occlusal surface images under different enhancement factor *α* values.

**Figure 5:** Proposed dental restoration network: (a) generator network; (b) global discriminator network; and (c) local discriminator network. The global discriminator takes the entire occlusal surface image as input, while the local discriminator takes only a small region around the missing tooth as input. *Note. n* and *k* refer to number of feature maps and kernel size, respectively.

**Figure 6:** Dilated convolution layers are composed of four blocks of Conv.-BN-ReLU. *Note.* r and s refer to number of dilation rate and stride, respectively.

**Figure 7:** Example of a patient dentition with defects (#46) occurring at the first mandibular molar. The seagreen biomorphic structures (occlusal groove and occlusal fingerprint) of the occlusal surface are shown in the red boxes.

The article "A Dual Discriminator Adversarial Learning Approach for Dental Occlusal Surface Reconstruction" was published in 2022. Journal: J Healthc Eng.

**Figure 8:** Occlusal surface generation results. The third to fifth columns denote three restored teeth under various training stages. The extracted occlusal fingerprint (in yellow box) and occlusal groove (in red box) are similar to the targets.

**Figure 9:** Training loss versus training iterations.

**Figure 10:** Standard box plots of different enhancement factors, in terms of PSNR, FSIM, and SSIM.

**Figure 11:** Ablation studies of the different convolutional layers. The first column provides a sample with the goldenrod color representing the defective region to be repaired. The second column provides the corresponding ground truth sample. The third to fourth columns provide a comparison between two convolutions and the deviation analysis of the occlusal surface.

**Figure 12:** Qualitative comparisons of three occlusal surface samples.

**Figure 13:** One real-world dental crown prosthesis: (a) the occlusal fingerprint distribution of the dental crown (#36) designed by our method and the contralateral tooth (#46) and (b) the dental crown designed by dentist.

**Figure 14:** Boxplots for deviation measurements.

**Algorithm 1:** Standardized processing of the dental model posture.

**Algorithm 2:** Depth map calculation.

**Table 1:** Average results in terms of three quality metrics. Note: values are denoted as mean ± standard deviation.

Metric	PSNR ↑	FSIM ↑	SSIM ↑
Stage I	27.833 ± 0.336	0.961 ± 0.016	0.933 ± 0.014
Stage II	28.129 ± 0.274	0.967 ± 0.012	0.948 ± 0.009
Stage III	34.264 ± 1.228	0.993 ± 0.008	0.985 ± 0.005

**Table 2:** Average results in terms of three quality metrics.

Metric	PSNR ↑	FSIM ↑	SSIM ↑
Pix2pix [25]	28.352 ± 1.891	0.961 ± 0.014	0.953 ± 0.011
CrownDesNet [24]	28.917 ± 2.248	0.975 ± 0.009	0.966 ± 0.012
Dental-GAN [27]	30.133 ± 2.099	0.976 ± 0.017	0.968 ± 0.014
DAIS [10]	31.454 ± 1.708	0.982 ± 0.013	0.974 ± 0.010
GL-GAN [34]	29.705 ± 2.419	0.973 ± 0.011	0.968 ± 0.016
DentalRecNet	34.264 ± 1.228	0.993 ± 0.008	0.985 ± 0.005

## Data Availability

The data used to support the findings of this study are available from the corresponding author upon request.

## References

[1] Tian S., Dai N., Cheng X., Li L., Sun Y., Cui H. (2019). Relative trajectory-driven virtual dynamic occlusal adjustment for dental restorations. *Medical, & Biological Engineering & Computing*.

[2] Chung M., Lee J., Song W. (2020). Automatic registration between dental cone-beam ct and scanned surface via deep pose regression neural networks and clustered similarities. *IEEE Transactions on Medical Imaging*.

[3] Machoy M., Seeliger J., Szyszka-SommerfeldMonika L. (2017). The use of optical coherence tomography in dental diagnostics: a state-of-the-art review. *Journal of Healthcare Engineering*.

The article "A Dual Discriminator Adversarial Learning Approach for Dental Occlusal Surface Reconstruction" was published in 2022. Journal: J Healthc Eng.

[4] Charlson F. J., Ferrari A. J., Santomauro D. F. (2018). Global epidemiology and burden of schizophrenia: findings from the global burden of disease study 2016. *Schizophrenia Bulletin*.

[5] Tribst J. P. M., Dal Piva A. M. d. O., Lo Giudice R. (2020). The influence of custom-milled framework design for an implant-supported full-arch fixed dental prosthesis: 3D-FEA study. *International Journal of Environmental Research and Public Health*.

[6] Ausiello P., Ciaramella S. (2019). Adhesive class I restorations in sound molar teeth incorporating combined resin-composite and glass ionomer materials: CAD-FE modeling and analysis. *Dental Materials*.

[7] Penteado M. M., Tribst J. P. M., Dal Piva A. M. (2019). Mechanical behavior of conceptual posterior dental crowns with functional elasticity gradient. *American Journal of Dentistry*.

[8] Kantardžić I., Vasiljević D., Lužanin O., Maravić T., Blažić L. (2018). Influence of the restorative procedure factors on stress values in premolar with MOD cavity: a finite element study. *Medical, & Biological Engineering & Computing*.

[9] Yuan T., Wang Y., Hou Z., Wang J. (2020). Tooth segmentation and gingival tissue deformation framework for 3D orthodontic treatment planning and evaluating. *Medical, & Biological Engineering & Computing*.

[10] Tian S., Wang M., Yuan F. (2021). Efficient computer-aided design of dental inlay restoration: a deep adversarial framework. *IEEE Transactions on Medical Imaging*.

[11] Fan R., Jin X. (2014). Tooth shape restoration with template feature line matching. *Journal of Computer Aided Design and Computer Graphics*.

[12] Zhang C., Liu T., Liao W., Yang T., Jiang L. (2017). Computer-aided design of dental inlay restoration based on dual-factor constrained deformation. *Advances in Engineering Software*.

[13] Li X., Wang X., Chen M. (2018). Accurate extraction of outermost biological characteristic curves in tooth preparations with fuzzy regions. *Computers in Biology and Medicine*.

[14] Liu L., Xu J., Huan Y., Zou Z., Yeh S.-C., Zheng L.-R. (2020). A smart dental health-iot platform based on intelligent hardware, deep learning, and mobile terminal. *IEEE Journal of Biomedical and Health Informatics*.

[15] Wu C.-H., Tsai W.-H., Chen Y.-H., Liu J.-K., Sun Y.-N. (2018). Model-based orthodontic assessments for dental panoramic radiographs. *IEEE Journal of Biomedical and Health Informatics*.

[16] Lai Y., Fan F., Wu Q. (2021). LCANet: learnable connected attention network for human identification using dental images. *IEEE Transactions on Medical Imaging*.

[17] Cheng B., Wang W. (2019). Dental hard tissue morphological segmentation with sparse representation-based classifier. *Medical, & Biological Engineering & Computing*.

The article "A Dual Discriminator Adversarial Learning Approach for Dental Occlusal Surface Reconstruction" was published in 2022. Journal: J Healthc Eng.

[18] Xiao D., Lian C., Deng H. (2021). Estimating reference bony shape models for orthognathic surgical planning using 3D point-cloud deep learning. *IEEE Journal of Biomedical and Health Informatics*.

[19] Hatvani J., Basarab A., Tourneret J.-Y., Kouame M., Kouamé D. (2019). A tensor factorization method for 3-D super resolution with application to dental CT. *IEEE Transactions on Medical Imaging*.

[20] Lee J.-H., Kim D.-H., Jeong S.-N., Choi S.-H. (2018). Detection and diagnosis of dental caries using a deep learning-based convolutional neural network algorithm. *Journal of Dentistry*.

[21] Moran M. B. H., Faria M. D. B., Giraldi G. A., Bastos L. F., Conci A. (2021). Using super-resolution generative adversarial network models and transfer learning to obtain high resolution digital periapical radiographs. *Computers in Biology and Medicine*.

[22] Lian C., Wang L., Wu T. H. (2020). Deep multi-scale mesh feature learning for automated labeling of raw dental surfaces from 3D intraoral scanners. *IEEE Transactions on Medical Imaging*.

[23] Torosdagli N., Liberton D. K., Verma P. (2018). Deep geodesic learning for segmentation and anatomical landmarking. *IEEE Transactions on Medical Imaging*.

[24] Hwang J.-J., Azernikov S., Efros A. A., Yu S. X. (2018). *Learning beyond Human Expertise with Generative Models for Dental Restorations*.

[25] Isola P., Zhu J.-Y., Zhou T., Efros A. A. (2017). Image-to-image translation with conditional adversarial networks. *Proceedings of the IEEE Conference on Computer Vision and Pattern Recognition (CVPR)*.

[26] Yuan F., Dai N., Tian S. (2020). Personalized design technique for the dental occlusal surface based on conditional generative adversarial networks. *International Journal for Numerical Methods in Biomedical Engineering*.

[27] Fezza S. A., Larabi M., Faraoun K. M. (2014). Stereoscopic image quality metric based on local entropy and binocular just noticeable difference. *Proceedings of the IEEE International Conference on Image Processing*.

[28] Chen Y., Liu L., Tao J. (2021). The improved image inpainting algorithm via encoder and similarity constraint. *The Visual Computer*.

[29] Xia W., Yang Y., Xue J.-H., Wu B. (2021). TediGAN: text-Guided diverse face image generation and manipulation. *Proceedings of the IEEE Conference On Computer Vision And Pattern Recognition*.

[30] Chen Y., Zhang H., Liu L. (2021). Research on image inpainting algorithm of improved total variation minimization method. *Journal of Ambient Intelligence and Humanized Computing*.

[31] Chen Y., Liu L., Tao J. (2021). The image annotation algorithm using convolutional features from intermediate layer of deep learning. *Multimedia Tools and Applications*.

The article "A Dual Discriminator Adversarial Learning Approach for Dental Occlusal Surface Reconstruction" was published in 2022. Journal: J Healthc Eng.

[32] Chen Y., Liu L., Phonevilay V. (2021). Image super-resolution reconstruction based on feature map attention mechanism. *Applied Intelligence*.

[33] Xu J., Wan C. (2021). A novel multi-modal fundus image fusion method for guiding the laser surgery of central serous chorioretinopathy. *Mathematical Biosciences and Engineering*.

[34] Iizuka S., Simo-Serra E., Ishikawa H. (2017). Globally and locally consistent image completion. *ACM Transactions on Graphics*.

[35] Li Y., Liu S., Yang J., Yang M.-H. (2017). Generative face completion. *Proceedings of the IEEE Conference On Computer Vision And Pattern Recognition*.

[36] Kong Z., Li T., Luo J., Xu S. (2019). Automatic tissue image segmentation based on image processing and deep learning. *Journal of Healthcare Engineering*.

[37] Song Q., Zhao L., Luo X., Dou X. (2017). Using deep learning for classification of lung nodules on computed tomography images. *Journal of Healthcare Engineering*.

[38] Yang Q., Yan P., Zhang Y. (2018). Low-dose ct image denoising using a generative adversarial network with wasserstein distance and perceptual loss. *IEEE Transactions on Medical Imaging*.

[39] Abadi M., Agarwal A., Barham P. (2016). *Tensorflow: Large-Scale Machine Learning on Heterogeneous Distributed Systems*.

[40] Luo Y., Chen K., Liu L. (2020). Dehaze of cataractous retinal images using an unpaired generative adversarial network. *IEEE Journal of Biomedical and Health Informatics*.

[41] Dar S. U., Yurt M., Karacan L., Erdem A., Erdem E., Cukur T. (2019). Image synthesis in multi-contrast mri with conditional generative adversarial networks. *IEEE Transactions on Medical Imaging*.

[42] Zhang J., Xia J. J., Li J., Zhou X. (2017). Reconstruction-based digital dental occlusion of the partially edentulous dentition. *IEEE Journal of Biomedical and Health Informatics*.

[43] Sánchez Lasheras F., Gracia Rodríguez J., Mauvezín-Quevedo M. (2019). Does the transversal screw design increase the risk of mechanical complications in dental implants? A finite elements analysis. *International Journal for Numerical Methods in Biomedical Engineering*.

[44] Fiorenza L., Nguyen H. N., Benazzi S. (2015). Stress distribution and molar macrowear in pongo pygmaeus: a new approach through finite element and occlusal fingerprint analyses. *Human Evolution*.

[45] Nauata N., Chang K.-H., Cheng C.-Y., Mori G., Furukawa Y., House-Gan (2020). House-GAN: relational generative adversarial networks for graph-constrained house layout generation, Computer Vision - ECCV 2020. *Proceedings of the European Conference on Computer Vision*.

The article "A Dual Discriminator Adversarial Learning Approach for Dental Occlusal Surface Reconstruction" was published in 2022. Journal: J Healthc Eng.

[46] Zhai M., Chen L., Mori G. (2021). Hyper-LifelongGAN: scalable lifelong learning for image conditioned generation. *Proceedings of the IEEE Conference on Computer Vision and Pattern Recognition*.

